The article "Trypanosoma brucei centrin5 is enriched in the flagellum and interacts with other centrins in a calcium‐dependent manner" was published in 2019. Journal: FEBS Open Bio.

# *Trypanosoma brucei* centrin5 is enriched in the flagellum and interacts with other centrins in a calcium‐dependent manner

**DOI:** 10.1002/2211-5463.12683

**Published:** 2019-07-09

**Authors:** Fangzhen Shan, Xiao Yang, Yating Diwu, Haoyu Ma, Xiaoming Tu

**Affiliations:** ^1^ Hefei National Laboratory for Physical Science at Microscale and School of Life Science University of Science and Technology of China Hefei China

**Keywords:** Ca^2+^ ions binding, protein interactions, TbCentrin5, *Trypanosoma brucei*

## Abstract

Centrin is an evolutionarily conserved EF‐hand‐containing protein, which is present in eukaryotic organisms as diverse as algae, yeast, and humans. Centrins are associated with the microtubule‐organizing center and with centrosome‐related structures, such as basal bodies in flagellar and ciliated cells, and the spindle pole body in yeast. Five centrin genes have been identified in *Trypanosoma brucei* (*T. brucei*), a protozoan parasite that causes sleeping sickness in humans and nagana in cattle in sub‐Saharan Africa. In the present study, we identified that centrin5 of *T. brucei* (TbCentrin5) is localized throughout the cytosol and nucleus and enriched in the flagellum. We further identified that TbCentrin5 binds Ca^2+^ ions with a high affinity and constructed a model of TbCentrin5 bound by Ca^2+^ ions. Meanwhile, we observed that TbCentrin5 interacts with TbCentrin1, TbCentrin3, and TbCentrin4 and that the interactions are Ca^2+^‐dependent, suggesting that TbCentrin5 is able to form different complexes with other TbCentrins to participate in relevant cellular processes. Our study provides a foundation for better understanding of the biological roles of TbCentrin5.

**Abbreviations**
CaM: calmodulin
CTD: C‐terminal domain
DAPI: 4',6‐diamidino‐2‐phenylindole
ITC: isothermal titration calorimetry
NTD: N‐terminal domain
RT‐PCR: reverse transcription‐PCR
TnC: troponin

Centrins are a member of the EF‐hand calmodulin (CaM) superfamily, which are highly conserved in eukaryotic cells. Centrins were initially identified in unicellular green algae 1, as the essential components of basal bodies‐associated and Ca^2+^‐sensitive contracting fibers. Subsequently, homologous centrin proteins were observed in the microtubule‐organizing center 2, 3, 4, 5. The functions of centrins were diverse in the cellular processes, including spindle pole body duplication 4, cellular morphogenesis 6, nucleotide excision repair 7, mRNA export 8, and protein degradation 9. In green algae, the flagellar contraction is regulated by contractile fibers containing centrin and the contraction depending on the increase in intracellular concentration of Ca^2+^ ions 1, 10, suggesting that centrin is responsible for Ca^2+^‐dependent cell motility. Target Sfi1 in yeast and its homologous protein (hSfi1) in humans were identified to interact centrins and responsible for SPB duplication 11, 12. In humans, two centrins (HsCentrin1 and HsCentrin2) with high sequence identity are involved in the centrosome/basal body segregation, ciliary beating, and mRNA and protein export 2, 3, 13, 14, 15. HsCentrin3 is involved in centrosome/basal body duplication 16, 17.

The article "Trypanosoma brucei centrin5 is enriched in the flagellum and interacts with other centrins in a calcium‐dependent manner" was published in 2019. Journal: FEBS Open Bio.

The overall topology of centrins or centrin/target peptide complexes reported by NMR spectroscopy or X‐ray crystallography 6, 11, 18, 19, 20, 21 is highly conserved and similar to CaM and troponin (TnC). The structure of centrin generally contains four EF‐hands comprised of seven to eight α‐helices. The structure of centrin can be divided into two independent domains, N‐terminal domain (NTD) and C‐terminal domain (CTD). Each domain contains a pair of EF‐hands. The two domains are linked by a loop or a long α‐helix and form a dumbbell structure. In all structures of centrins except *Mus musculus* Centrin1 (MmCentrin1) 19 and *Chlamydomonas* *reinhardtii* centrin (CrCentrin) 22, the two EF‐hands of CTD instead of all the four EF‐hands can be saturated by Ca^2+^ ions. The highly conserved CTD shows a higher affinity with Ca^2+ ^ions and other partners 11, 23, 24. Meanwhile, NTD containing unconserved and unstructured 20–25 residues at the front shows a lower affinity with Ca^2+^ ions and its partners 11, 20. Compared with CaM and TnC, the extended 20–25 residues in the NTD may have specialized biological function that is metal ion‐dependent during self‐assembly of centrin 25, 26.

In *Trypanosoma brucei* (*T. brucei*), a protozoan parasite that causes sleeping sickness in humans and nagana in cattle in sub‐Saharan Africa, five centrin isoforms have been identified 27, 28. TbCentrin1 (Tb927.04.2260) and TbCentrin2 (Tb927.08.1080) are localized to the basal body and are essential for basal body duplication 27. TbCentrin3 (Tb927.10.8710) is localized in the flagellum and is required for the flagellar motility 29. TbCentirn4 (Tb927.07.3410) is localized to both the basal bodies and the bilobe structure and is involved in organelle segregation and the coordination between karyokinesis and cytokinesis 30, 31. The role of centrin5 of *T. brucei* (TbCentrin5; Tb927.11.13900) is still unknown.

Here, we investigated the localization of TbCentrin5 in *T. brucei* and identified the interactions between TbCentrin5 and Ca^2+ ^ions. We further identified that TbCentrin5 is able to interact with other TbCentrins and the interactions are Ca^2+^‐dependent. The work will provide a basis for better understanding of the biological functions of TbCentrin5.

The article "Trypanosoma brucei centrin5 is enriched in the flagellum and interacts with other centrins in a calcium‐dependent manner" was published in 2019. Journal: FEBS Open Bio.

## Materials and methods

### Phylogenetic analyses of centrin protein sequences

The centrin protein sequences of *T. brucei* were obtained from TriTrypDB (https://tritrypdb.org/tritrypdb/). All other centrin protein sequences were obtained from NCBI protein database (https://www.ncbi.nlm.nih.gov/protein) and UniProt (https://www.uniprot.org/). Sequences were aligned using clustalx 32 with default alignment parameters. The sequence trees were reconstructed with Neighbor‐Joining algorithm using mega7 33. Bootstrap analysis (> 70, based on 500 replicates) provided a confidence measure for the detected relationships of branches in the phylogenetic tree.

### Cell culture

The wild‐type procyclic Lister 427 strain was cultivated at 28 °C in Cunningham's medium supplemented with 10% FBS. The procyclic 29‐13 strain 34 was cultivated at 28 °C in Cunningham’s medium containing 10% FBS, supplemented with 15 μg·mL^−1^ G418 and 50 μg·mL^−1^ hygromycin.

### RNA interference

RNA interference (RNAi) of TbCentrin5 was performed using the RNAi vector pZJM. Recombinant pZJM vector containing segment (nucleotide number 121–420) of TbCentrin5 was linearized and electroporated into *T. brucei* procyclic forms from 427 strain. The transfection by electroporation was carried out as follows: Briefly, 10^8^ cells were harvested and washed twice with cytomix buffer (120 mm KCl, 0.15 mm CaCl_2_, 10 mm K_2_HPO_4_, 10 mm KH_2_PO_4_, 25 mm Hepes, 2 mm EGTA, 5 mm MgCl_2_, 2 mm ATP, 5 mm glutathione, pH 7.6) and suspended in 0.45 mL of cytomix buffer containing 30 μg of the linearized vectors. Electroporation was carried out in a 2‐mm cuvette (Bio‐Rad, Berkeley, CA, USA) using the Gene Pulser (BTX ECM630, Holliston, MA, USA) with parameters set as follows: 2.0 kV voltages, 25 μF capacitance, and 200 Ω resistance. The transfected cells were immediately transferred into 10 mL of fresh Cunningham’s medium. Transfectants were selected with 10 μg·mL^−1^ zeocin and were induced with 1.0 μg·mL^−1^ tetracycline.

### *In situ* epitope tagging of endogenous proteins

For *in situ* tagging of TbCentrin5, the cDNA segment (nucleotide number 121–558) was cloned into pC‐EYFP‐NEO vector 35. The recombinant vectors were linearized and electroporated into *T. brucei* procyclic forms from 427 strain. The transfection conditions were the same described as above. Successful transfectants were selected under 2.5 μg·mL^−1^ G418. Expression of TbCentrin5‐EYFP fusion protein was verified by western blotting.

### Immunofluorescence microscopy

Cells stably expressing TbCentrin5‐EYFP were harvested and washed twice with PBS. Resuspended cells were fixed with 4% paraformaldehyde and washed with PBS. Fixed cells were settled on the coverslip at room temperature for 30 min. The cells were stained with 4′,6‐diamidino‐2‐phenylindole (DAPI) and examined with an inverted microscope (Model IX73; Olympus, Tokyo, Japan). Images were analyzed by imagej (NIH, Bethesda, MD, USA).

The article "Trypanosoma brucei centrin5 is enriched in the flagellum and interacts with other centrins in a calcium‐dependent manner" was published in 2019. Journal: FEBS Open Bio.

### Protein expression and purification

Full‐length gene encoding TbCentrin5 was amplified by PCR from the genomic DNA of *T. brucei* and cloned into a modifier vector pET‐28a (+) (Novagen, Darmstadt, Germany), which provided a cut site of TEV protease at the N terminus to remove His‐tag. The recombinant vector was transformed into *Escherichia coli* BL21 (DE3). The transformed cells were cultured in LB at 37 °C until OD_600_ reached 0.8 and induced by 0.5 mm IPTG at 16 °C for 20 h. The cells were harvested and purified in lysis buffer containing 20 mm Tris and 500 mm NaCl at pH 7.0. The eluted protein was digested by TEV protease and further purified by gel filtration column Sephadex G‐75 (GE Healthcare, Chicago, IL, USA).

### Structure modeling

The 3D structure of TbCentrin5 or the complex of TbCentrin5 and Ca^2+ ^ions was carried out using SWISS‐MODEL based on homology modeling techniques 36. The evolutionarily related protein structures were searched as templates based on the amino acid sequence of TbCentrin5. More than five hundred templates were searched and estimated by Global model quality estimate (GMQE) 37 and quaternary structure quality estimate (QSQE) 38. Top‐ranked templates were selected as templates for building model automatically. The model was finally evaluated and optimized by pairwise distance constraints that represented ensemble information from all template structures found.

### Isothermal titration calorimetry

Isothermal titration calorimetry (ITC) measurements were performed on iTC200 (GE Healthcare) at 16 °C to investigate the Ca^2+^‐binding capacity and the interactions between TbCentrin5 and TbCentrin1/2/3/4. Samples of TbCentrin5 titrated with Ca^2+ ^ions were mixed with EGTA to remove potential Ca^2+^ ions and then further purified by gel filtration column Sephadex G‐75 (GE Healthcare). TbCentrin5 and calcium ions were equilibrated in the same buffer containing 20 mm Tris/HCl (pH 7.0) and 100 mm NaCl. 0.1 mm TbCentrin5 in cell was titrated against 2.0 mm CaCl_2_ from syringe. Two microliter of CaCl_2_ was injected into 0.2 mL TbCentrin5 at 120 s intervals. Samples of TbCentrin1/2/3/4 titrated with TbCentrin5 were purified and equilibrated as above expect mixed with EGTA or not. Fifty micromolar TbCentrin1/2/3/4 in the cell was titrated against 0.5 mm TbCentrin5 from the syringe with the same sample volume and rotate speed. The data collected were analyzed by microcal LLC ITC software (MicroCal, Malvern, UK).

The article "Trypanosoma brucei centrin5 is enriched in the flagellum and interacts with other centrins in a calcium‐dependent manner" was published in 2019. Journal: FEBS Open Bio.

### Sedimentation assay

Sedimentation assay was carried out according to the procedures published previously 29. In brief, the wild‐type 29‐13 cell line, the noninduced control cells, and TbCentrin5 RNAi cells after tetracycline induction for 3 days were each suspended to ~ 5×10^6^ cells·mL^−1^ in fresh medium. Each cell line was cultured in two cuvettes and incubated at 26 °C and was measured by optical density (600 nm) every 2 h. To monitor the OD_600_, one cuvette was resuspended for monitoring cell growth while the other cuvette was not disturbed for monitoring sedimentation. The change in the OD_600_ (ΔOD_600_) was calculated by subtracting the OD_600_ of the resuspended sample from that of the undisturbed sample. The experiment was repeated three times.

## Results and Discussion

### Phylogenetic analysis of TbCentrin5

To further understand the position of TbCentrin5 in evolution and its relationship with other centrins that have been identified in other organisms, a phylogenetic analysis was performed using a Neighbor‐Joining method (Fig. 1A). Because the sequences of centrins are conserved, Neighbor‐Joining method was selected. The presence of sequences of centrins from animal, fungi, and protist in this evolutionary tree indicates that those centrins come possibly from an ancestral protein in eukaryotic evolution. In the evolutionary tree, centrins from *T. brucei* are on different branches with centrins from higher animal, but closer to centrins from fungi and other protest, especially to centrins from *Leishmania major* (*L. major*) which belong to the same family of *Trypanosomatidae* as *T. brucei*. TbCentrin5 and TbCentrin2 were on utterly different branches with other centrins but same as LmCentrin4 and LmCentrin3, suggesting that TbCentrin5 and TbCentrin2 are far from other centrins but closer to LmCentrin4 and LmCentrin3. The phylogenetic analysis indicated the position of TbCentrin5 and its relationship with other centrins, which is helpful for us to determine the location of *Trypanosoma* genera in the evolution.

**Figure 1:** Characterization of TbCentrin5. (A) Evolutionary tree of centrins. Numbers on branches represent bootstrap support values. Hs, *Human sapiens*; Mm, *Mus musculus*; Cr, *Chlamydomonas_reinhardtii*; Tg, *Toxoplasma gondii*; Eo, *Euplotes octocarinatus*; Sd, *Scherffelia dubia*; Sc, *Saccharomyces_cerevisiae*; Tt, *Tetrahymena thermophila*; Ld, *Leishmania donovani*; Lm, *Leishmania major*; Tb, *Trypanosoma brucei*; (B) The expression of TbCentrin5‐EYFP examined by western blot with anti‐GFP probe. The levels of α‐tubulin served as the loading control. (C) The subcellular localization of TbCentrin5. The localization of TbCentrin5‐EYFP (green) was examined in paraformaldehyde‐fixed intact cells. Cells were stained DAPI for DNA (blue), small blue dots are kinetoplasts, and large blue structures are nuclei. 1N1K, 1N2K, and 2N2K cells were tabulated, respectively. Scale bars: 5 μm.

The article "Trypanosoma brucei centrin5 is enriched in the flagellum and interacts with other centrins in a calcium‐dependent manner" was published in 2019. Journal: FEBS Open Bio.

### TbCentrin5 is localized throughout the cytosol and nucleus and enriched in the flagellum

To determine the subcellular localization of TbCentrin5, TbLa was endogenously tagged with EYFP at the C terminus. The level of TbCentrin5‐EYFP fusion protein was examined by western blot with GFP probe, which indicated the successful expression of TbCentrin5‐EYFP *in vivo* (Fig. 1B). Fluorescence microscopy demonstrated that TbCentrin5‐EYFP appeared to spread throughout the cell and was enriched in flagellum (Fig. 1C). Intriguingly, the localization of TbCentrin5 in nucleus changed through the cell cycle. In the early stage (1N1K) of the cell cycle, TbCentrin5 was slightly distributed in nucleus. As the cell cycle progressed (1N2K and 2N2K), the distribution of TbCentrin5 in nucleus became stronger. The results suggested that TbCentrin5 might be involved in the karyokinesis.

### Sequence analysis of TbCentrin5

The sequence of TbCentrin5 was aligned with other centrins from *T. brucei, L. major *and* Homo sapiens* using clustalw2 and espript 3.0 32, 39. TbCentrin5 shares about 29%, 33%, 27%, 31%, 38%, and 45% sequence identity with TbCentrin1‐4, HsCentrin1, and LmCentrin2, respectively (Fig. 2). The result of sequence alignment also verified the credibility of the evolutionary tree in Fig. 1A. Although the structures of centrins are conserved 6, 11, 18, 19, 20, 21, the sequences of centrins show diversity. Especially, the sequences of the first ~ 25 residues at the N terminus show diverse length and very low similarity. In contrast with CaM and TnC, the extended ~ 25 amino acids at the N terminus of centrins display diversity in length and sequence, indicating that centrins may have more versatile functions than CaM and TnC.

**Figure 2:** Multiple sequence alignments of TbCentrin5 with other centrins. Tb, *Trypanosoma brucei*; Hs, *Homo sapiens*; Lm, *Leishmania major*. Identical residues are shaded in red box, and conserved residues are colored in red.

### Structure modeling of TbCentrin5

To better understand the functions of TbCentrin5, the model of TbCentrin5 was built using SWISS‐MODEL 36, which builds model based on homology modeling techniques. Because the first 25 amino acids of TbCentrin5 show low conservation, the sequence of TbCentrin5 without the first 25 amino acids was placed for modeling. A total of 4015 templates were found from template library extracted from the PDB 40 to match the sequence of TbCentrin5, and five templates were selected for modeling. The quality of model built by SWISS‐MODEL is rapidly reduced when sequence identity is below ~ 30% and is reliable when sequence identity is more than ~ 40% 41, 42. Finally, MmCentrin1 (PDB: 5d43), HsCentrin2 (PDB: 2ggm), SdCentrin (PDB: 3kf9), and CrCentrin (PDB: 3qrx) with respective sequence identity of 43%, 42%, 41%, and 39% were selected to build model (Fig. 3). The scores of the model estimated by GMQE and QSQE were 0.64 and −1.23, respectively. In addition, the analysis of Ramachandran plots showed that 96% of the residues are in the most favored region (Fig. 4). The evaluation indicated that the model is of high quality and reliable. The structure model of TbCentrin5 is comprised of four EF‐hands containing seven α‐helices. Interestingly, a very short α‐helix was formed in the loop of EF‐hand IV because the loop is longer than that in general EF‐hand. TbCentrin5 is divided into NTD and CTD by the long α4 and adopts a shape like a dumbbell.

The article "Trypanosoma brucei centrin5 is enriched in the flagellum and interacts with other centrins in a calcium‐dependent manner" was published in 2019. Journal: FEBS Open Bio.

**Figure 3:** Structure model of TbCentrin5. The model was built by SWISS‐MODEL based on homology modeling techniques.

**Figure 4:** The model of TbCentrin5 was evaluated by Ramachandran plots.

### Purification of TbCentrin5

Centrin5 of *T. brucei* was expressed and purified as described above. The elution volume of TbCentrin5 from Superdex G‐75 column is approximate 66 mL, which corresponds to a molecular weight about 36 kDa (Fig. 5A). The calculated molecular weight of TbCentrin5 containing 186 amino acids is about 20 kDa. In addition, SDS/PAGE indicated no disulfide bond formation of the purified TbCentrin5 proteins, which suggested TbCentrin5 was expressed and purified as a homodimer.

**Figure 5:** The Ca^2+^ binding of TbCentrin5. (A) Gel filtration of Superdex G‐75 column and SDS/PAGE analysis of TbCentrin5. (B) Saturated titration of TbCentrin5 with Ca^2+^ ions was measured by ITC. (C) The model of TbCentrin5 bound by Ca^2+^ ions. Ca^2+^‐binding site at the loop of EF‐hand III (D) and EF‐hand IV (E). Cyan‐colored sticks represent the residues which interact with Ca^2+^ ions, red represents oxygen atom, blue represents nitrogen atom. Magenta lines represent coordinated bonds.

### TbCentrin5 binds to Ca^2+^ ions with a high affinity

As an important second messenger, Ca^2+^ ion is involved in many biological regulation processes 43. ITC was performed to investigate the Ca^2+^‐binding property of TbCentrin5 (Fig. 5B). The result showed that TbCentrin5 (pretreated with EDTA) binds to Ca^2+^ ions with a high affinity (*K*_d_ = 4.8 μm) in an exothermic mode and one molecule of TbCentrin5 is able to bind two Ca^2+^ ions (*N* = 2).

The article "Trypanosoma brucei centrin5 is enriched in the flagellum and interacts with other centrins in a calcium‐dependent manner" was published in 2019. Journal: FEBS Open Bio.

The Ca^2+^‐binding mode of TbCentrin5 is similar to that of TbCentrin4 21, HsCentrin2 20, 44, and ScCdc31 11 where one centrin molecule binds two Ca^2+ ^ions. In other Ca^2+^‐binding modes, one centrin molecule binds more than two Ca^2+^ ions 19, 22. Because of the higher binding affinity of CTD of centrins compared with NTD, CTD was preferentially saturated with Ca^2+^ ions 11, 20, 23, 24. Therefore, the Ca^2+^‐binding site of TbCentrin5 should be located in the CTD containing EF‐hand III and EF‐hand IV. The structure model of TbCentrin5 bound by Ca^2+^ ions was built using SWISS‐MODEL (Fig. 5C). As a Ca^2+^‐binding motif, EF‐hand contains the specific amino acid sequences (Table 1) 45 that provide carboxyl oxygen atoms for coordinating Ca^2+^ ions. The residues (Asp117, Tyr123, Asp128) in the loop of EF‐hand III may provide five coordinated bonds for Ca^2+^ ions binding (Fig. 5D). The conformation of EF‐hands may change due to the binding of Ca^2+^ ions to EF‐hands, resulting in the change of the direction of Lys121, which may also provide a coordinated bond for Ca^2+^ ions binding. The loop of EF‐hand IV in TbCentrin5 is longer than its counterparts in other centrins (Fig. 2), resulting in the change of the location of the residues that provide coordinated bonds for Ca^2+^ ions binding. The residues (Pro154, Asp162, Thr170, Glu175) in the loop of EF‐hand IV may provide six coordinated bonds for Ca^2+^ ions binding (Fig. 5E). The residues in the EF‐hand III and EF‐hand IV have the ability to provide sufficient coordinated bonds for Ca^2+^ ions binding, indicating TbCentrin5 has a high Ca^2+^‐binding affinity and forms a stable complex with Ca^2+^ ions.

**Table 1:** The sequence preference of the loop in EF‐hand. bb, backbone; sc, side chain.

EF‐hand loop position	1	2	3	4	5	6	7	8	9	10	11	12
Coordinated ligand	X sc		Y sc		Z sc		−Y bb		−X sc^a^			−Z sc2
Most common	Asp 100%	Lys 29%	Asp 76%	Gly 56%	Gly 56%	Gly 96%	Thr 23%	Ile 68%	Asp 32%	Phe 23%	Glu 29%	Glu 92%
Other frequently observed		Ala Gln Thr Val Ile Ser Glu Arg	Asn	Lys Arg Asn	Ser Asn		Phe Lys Gln Tyr Glu Arg	Val Leu	Ser Thr Glu Asn Gly Gln	Tyr Ala Thr Leu Glu Lys	Asp Lys Ala Pro Asn	Asp

a The ligand typically provided by a water molecule that is hydrogen‐bonded to the side chain of the residues at position 9.

### TbCentrin5 interacts with other centrins depending on Ca^2+ ^ions binding

In *T. brucei*, five centrin isoforms have been identified 27, 28. We have previously reported that TbCentrin4 interacts with TbCentrin1, TbCentrin2, and TbCentrin5 21. To investigate the interactions between TbCentrin5 and other TbCentrins and further enrich the interaction network of centrins from *T. brucei*, GST‐pull down assay and ITC were performed.

The article "Trypanosoma brucei centrin5 is enriched in the flagellum and interacts with other centrins in a calcium‐dependent manner" was published in 2019. Journal: FEBS Open Bio.

GST‐fused TbCentrin1‐4 and TbCentrin5‐HA were expressed and used in GST‐pull down assay (Fig. 6A). The results showed that TbCentrin5 interacts with TbCentrin1, TbCentrin3, and TbCentrin4 but not TbCentrin2.

**Figure 6:** Interactions between TbCentrin5 and other TbCentrins. (A) GST‐pull down assay. TbCentrin5‐3HA was pulled down by GST‐TbCentrin1‐4 and detected by western blot. ITCs of TbCentrin1‐4 titrated with TbCentrin5 were performed without (B) or with (C) EGTA treatment.

To further investigate the binding affinity of TbCentrin5 with TbCentrin1, TbCentrin3, and TbCentrin4, ITC analysis of TbCentrin1‐4 titrated with TbCentrin5 was carried out (Fig. 6B). The results verified the interactions between TbCentrin5 and TbCentrin1, 3, 4. The dissociation constants (*K*_d_ values) of TbCentrin5 binding to TbCentrin1, TbCentrin3, and TbCentrin4 are 105, 52, and 12 μm, respectively.

In the above experiments, EGTA was not added to remove the remaining Ca^2+^ ions in TbCentrins. In the protein expression in LB culture medium and purification procedures, Ca^2+^ ions may be copurified with TbCentrins. Therefore, it is necessary to ensure complete removal of Ca^2+^ ions by treatment of EGTA to investigate the effect of Ca^2+^ ions on the interactions between TbCentrin5 and other TbCentrins. ITC analysis of TbCentrin1, 2, 3, 4 titrated with TbCentrin5 was then performed without Ca^2+^ ions. In the absence of Ca^2+^ ions, TbCentrin5 is not able to interact with TbCentrin1, 2, 3, 4 (Fig. 6C). The results indicated that TbCentrin5 interacts with TbCentrin1, 3, 4 depending on Ca^2+^ ions binding. Binding to Ca^2+^ ions might induce the local conformational change of TbCentrin5, which results in the exposure of more hydrophobic region of TbCentrin5 to interact with other TbCentrins. Owing to these interactions, TbCentrin5 is able to form different complexes with other TbCentrins depending on cellular Ca^2+^ ions to participate in the relevant biological processes.

### Depletion of TbCentrin5 does not compromise the cell motility

To investigate whether depletion of TbCentrin5 impacts cell growth, RNAi targeting on TbCentrin5 was performed in procyclic 29‐13 cell line. Quantitative reverse transcription‐PCR (RT‐PCR) monitored that the mRNA level of TbCentrin5 in the RNAi cells decreased by ~ 80% compared with that in the noninduced control cells after tetracycline induction for 2 days (Fig. 7A). The result demonstrated that depletion of TbCentrin5 does not inhibit the cell growth significantly (Fig. 7A).

The article "Trypanosoma brucei centrin5 is enriched in the flagellum and interacts with other centrins in a calcium‐dependent manner" was published in 2019. Journal: FEBS Open Bio.

**Figure 7:** Sedimentation assays to monitor the cell motility. (A) Effect of TbCentrin5 RNAi on cell proliferation. Quantitative RT‐PCR was used to monitor the level of TbCentrin5 mRNA in noninduced control cells and RNAi cells (inset). (B) The parental 29‐13 cell line, the noninduced cells, and TbCentrin5 RNAi cells after tetracycline induction for 3 days were incubated in cuvettes. The change of cell density (ΔOD_600_) was determined and plotted against the time of incubation (hours). Three independent experiments were carried out, and the error bars represent SD.

TbCentrin5 has the same flagellum localization as TbCentrin3, and the effect of TbCentrin5 RNAi on cell growth is also similar to that of TbCentrin3 RNAi 29. It was reported that knockdown of TbCentrin3 compromised the cell motility 29. Therefore, the impact of knockdown of TbCentrin5 on the cell motility was also investigated. Sedimentation assay of cells after TbCentrin5 RNAi was performed. Monitored OD_600_ values among wild‐type 29‐13 cell line, the noninduced control cells, and TbCentrin5 RNAi cells showed no significant distinction (Fig. 7B). Under light microscopy, cells after the deficiency of TbCentrin5 did not display any unusual phenotype such as spinning and tumbling or losing motility compared with the noninduced control cells. The results indicated that the depletion of TbCentrin5 does not compromise the cell motility.

## Conclusion

In conclusion, we identified that TbCentrin5 is localized at the cytosol and nucleus and enriched in the flagellum. We further identified that TbCentrin5 binds Ca^2+ ^ions with a high affinity and built the model of TbCentrin5 bound by Ca^2+^ ions. Besides, we demonstrated that TbCentrin5 interacts with TbCentrin1, TbCentrin3, and TbCentrin4 depending on Ca^2+^ ions binding, suggesting TbCentrin5 might be able to form different complexes with other TbCentrins depending on cellular Ca^2+ ^ions to participate in the relevant biological processes. Our study will provide a basic information for better understanding the biological functions of TbCentrin5.

## Conflict of interest

The authors declare no conflicts of interest.

## Author contributions

FS and XT designed the research. FS, XY, YD, and HM performed the experiments. FS, XY, and XT analyzed the data. FS and XT wrote the paper. XY, YD, and HM discussed and gave suggestions on the manuscript.
